The article "Curative Effect of Prebiotics/Probiotics Preparations Combined with Zoledronic Acid + Calcitriol Regimen on Patients with Primary Osteoporosis and Their Influences on Bone Metabolism Markers" was retracted in 2024. Reasons: signs of a paper mill; suspected computer-generated content; unreliable results or conclusions; lack of ethics approval or compliance.

# Curative Effect of Prebiotics/Probiotics Preparations Combined with Zoledronic Acid + Calcitriol Regimen on Patients with Primary Osteoporosis and Their Influences on Bone Metabolism Markers

**DOI:** 10.1155/2022/3293362

**Published:** 2022-07-21

**Authors:** Ruipeng Jia, Ning Liu, Yanyan Zhu, Qiaoli Li

**Affiliations:** ^1^Department of Orthopaedic, Haikou People's Hospital, Haikou, Hainan 570208, China; ^2^Department of Orthopaedic, The 942nd Hospital of the PLA Joint Logistic Support Force, Yinchuan, Ningxia 750004, China; ^3^Department of Clinical Pharmacy, Ningbo Yinzhou No. 2 Hospital, Ningbo, Zhejiang 315000, China

## Abstract

**Objective:**

To explore the curative effect of prebiotics/probiotics preparations combined with zoledronic acid + calcitriol regimen on patients with primary osteoporosis (POP) and the influences of prebiotics/probiotics preparations combined with zoledronic acid + calcitriol regimen on markers of bone metabolism.

**Methods:**

126 elderly hospitalized patients with POP in our hospital from January 2020 to December 2021 were divided into the control group (*n* = 63) and the observation group (*n* = 63) by the random number table method. The patients in the control group were treated with zoledronic acid and calcitriol, while the patients in the observation group were additionally treated with prebiotics/probiotics preparations. The clinical curative effect, bone metabolism, calcium-phosphorus metabolism indexes, intestinal floras, and cytokines levels before and via treatment between the two groups were compared.

**Results:**

The total efficiency of the observation group was higher than that of the control group (*P* < 0.05). After treatment, the levels of bone gla protein (BGP), total propeptide of type I procollagen (PINP), and *β*-crosslaps (*β*-CTX) in both groups were lower than those before treatment, and the levels of BGP, total PINP, and *β*-CTX in the observation group were lower than those in the control group (*P* < 0.05). The levels of serum P in the both groups after treatment were lower than those before treatment, and the level of serum P in the observation group was lower than that in the control group (*P* < 0.05). The number of *Escherichia coli* after treatment in the two groups were less than that before treatment, and the number of *Escherichia coli* in the observation group was less than that in the control group (*P* < 0.05). The number of bifidobacteria and lactobacilli in the two groups after treatment were more than that before treatment, and the number of bifidobacteria and lactobacilli in the observation group were more than those in the control group (*P* < 0.05). After treatment, the levels of IL-6 and TNF-*α* in the two groups were lower than those before treatment, and the levels of IL-6 and TNF-*α* in the observation group was lower than those in the control group (*P* < 0.05). The levels of IGF-1 in the two groups after treatment were higher than those before treatment, and the levels of IGF-1 in the observation group was higher than that in the control group (*P* < 0.05).

The article "Curative Effect of Prebiotics/Probiotics Preparations Combined with Zoledronic Acid + Calcitriol Regimen on Patients with Primary Osteoporosis and Their Influences on Bone Metabolism Markers" was retracted in 2024. Reasons: signs of a paper mill; suspected computer-generated content; unreliable results or conclusions; lack of ethics approval or compliance.

**Conclusion:**

The response rate of prebiotics/probiotics preparations combined with zoledronic acid + calcitriol regimen is high in the treatment of POP patients, which ameliorates bone metabolism and intestinal floras, and suppresses cytokines release in patients with POP.

## 1. Introduction

Primary osteoporosis (POP) is a group of systemic bone illnesses primarily associated with increased bone fragility and easy fracture due to low mass, destruction of bone microarchitecture, and decreased bone strength. Nowadays, zoledronic acid, calcitriol, and other drugs are used in clinical treatment. Zoledronic acid is a diphosphate compound that specifically acts on bone, and it can inhibit bone resorption caused by increased osteoclast activity, thereby increasing bone density and enhancing bone strength [1]. However, related reports pointed out that some patients still have abnormal bone metabolism after zoledronic acid combined with calcitriol treatment [2]. At present, some studies have suggested that the occurrence and development of POP may be related to the abnormal intestinal flora [3]. Disturbance of intestinal flora can lead to decreased intestinal immunity, inhibit intestinal absorption of calcium and phosphorus, and affect bone health. Therefore, it may be possible to improve bone metabolism disorder by regulating intestinal flora. The bifidobacterium quadruple viable comprises four components of bifidobacterium, *Lactobacillus acidophilus*, *Enterococcus faecalis*, and *Bacillus cereus*. It can directly supplement normal physiological bacteria of human body, form biological barrier in intestinal tract, inhibit certain pathogenic bacteria in intestinal tract, promote intestinal peristalsis, adjust balance of intestinal flora, stimulate immunity of organism, participate in synthesis of vitamins, promote digestion and absorption of nutrients, and is the most commonly used medicine related to intestinal flora imbalance in clinical treatment. However, there are few reports on the treatment of POP by adjusting intestinal flora. Therefore, we want to explore the efficacy of prebiotic/probiotic preparations combined with zoledronic acid + calcitriol regimen in the treatment of POP patients and the effect on bone metabolism markers in this study.

## 2. Materials and Methods

### 2.1. Clinical Data

126 elderly hospitalized patients with POP in our hospital from January 2020 to December 2021 were included and randomly divided into the control group (group without prebiotics/probiotics preparations) and the observation group (group with prebiotics/probiotics preparations) by the random number table method, with 63 cases per group. In the control group, there were 22 males and 41 females; the average age was (72.52 ± 3.63) years; body weight (64.03 ± 4.45) kg; course of disease (5.17 ± 0.79) years. In the observation group, there were 39 females and 24 male; the average age was (72.49 ± 3.81) years; the body weight was (62.44 ± 5.11) kg; the course of disease was (5.20 ± 0.73) years old. The difference in the above data between the two groups was not markedly significant (*P* > 0.05).

The article "Curative Effect of Prebiotics/Probiotics Preparations Combined with Zoledronic Acid + Calcitriol Regimen on Patients with Primary Osteoporosis and Their Influences on Bone Metabolism Markers" was retracted in 2024. Reasons: signs of a paper mill; suspected computer-generated content; unreliable results or conclusions; lack of ethics approval or compliance.

### 2.2. Inclusion Criteria

(1) Meet the diagnostic criteria for POP in the Guidelines for the Diagnosis and Treatment of Primary Osteoporosis (2017) [4]; (2) all patients signed the informed consent; (3) age ≥ 60 years old.

### 2.3. Exclusion Criteria

(1) Patients who have severe kidney, liver, and heart diseases; (2) patients who have secondary osteoporosis; (3) patients who have tumor diseases; (4) patients with severe metabolic dysfunction; (5) those who are sensitive to the drugs used in this study; (6) patients with other inflammatory diseases; (7) patients with severe gastrointestinal diseases.

### 2.4. Methods

The control group was treated with zoledronic acid (Zhengda Tianqing Pharmaceutical Group, batch number: Guoyao Zhunzi H20041346, specifications: 5 ml: 4 mg) combined with calcitriol capsules (Zheng Haier Pharmaceutical Co. Ltd., batch number: Guoyao Zhunzi H20030491, specifications: 0.25 *μ*g *∗* 10 s), zoledronic acid 4 mg + 100 ml normal saline, intravenous infusion, instillation time over 15 min, a total of 1 injection. Calcitriol 1 tablet/time was taken after lunch, 1 time/d, for a total of 3 months of treatment.

On this basis, the control group was given Bifidobacterium quadruple viable tablets (Hangzhou Grand Bio-Pharmaceutical Co. Ltd., batch number: S20060010, specification: 0.5 g *∗* 24 s), 3 tablets/d, for a total of 3 months.

### 2.5. Observation Indicators

(1) Clinical efficacy: via treatment for 90 days, the clinical efficacy was evaluated according to the “Osteoporosis Identification, Diagnosis, and Treatment” [5]. Significant valid: the low back pain disappeared, the spinous process did not have percussion pain, the waist and knees were sore and weak, and the lower limbs. Weakness and other symptoms have been significantly improved, bone mineral density has increased by >2%, and activities are free. Effective: low back pain is significantly reduced; waist and knee soreness, lower extremity weakness, dizziness, and other symptoms are improved. The bone mineral density value is increased by ≤2%, and light work can be performed. Invalid: no improvement in clinical symptoms, limited daily life, and activities. (2) Bone metabolism index: collect 3 ml of fasting venous blood from patients, centrifuge at a rate of 3000 r/min, and after separating serum, use the chemiluminescence method to detect the osteocalcin (bone-*γ*) before treatment and after 3 months of treatment. The kit of Carboxyglutamic acid-containing protein, BGP, total collagen type 1 amino acid extension peptide (propeptide of type I procollagen, PINP), and *β*-collagen special sequence (*β*-crosslaps, *β*-CTX) levels, is provided by Roche. (3) Calcium and phosphorus metabolism: ELISA was used to detect serum Ca and P levels of patients before treatment and for 3 months after treatment. (4) Intestinal flora: take 0.5 g of fresh fecal samples from patients before treatment and 3 months after treatment, dilute it to 10-8 by the 10-fold dilution method, take 10 *μ*L of dilution for inoculation, and use the corresponding medium for cultivated at 37°C for 48 h, and counted the number of colonies after biochemical identification. (5) Cytokines: the radioimmunoassay was used to detect interleukin-6 (IL-6), tumor necrosis factor-*α* (TNF-*α*), and insulin-like growth factor-1 (IGF-1) levels, before treatment and 3 months after treatment.

The article "Curative Effect of Prebiotics/Probiotics Preparations Combined with Zoledronic Acid + Calcitriol Regimen on Patients with Primary Osteoporosis and Their Influences on Bone Metabolism Markers" was retracted in 2024. Reasons: signs of a paper mill; suspected computer-generated content; unreliable results or conclusions; lack of ethics approval or compliance.

### 2.6. Statistical Processing

We used the SPSS 22.0 software to process the date analysis, enumeration data were presented as (%), and differences between groups were compared by the *χ*^2^ test. The data in linear scale were presented as mean ± standard deviation (±*s*) after the normality test, and the independent *t*-test was used to compare differences between two groups, within-group differences were measured by paired A sample *t*-test. *P* < 0.05 indicates statistically significant difference.

## 3. Results

### 3.1. Comparison of Therapeutic Effects among Groups with/without Prebiotics/Probiotics Preparations

The total efficiency of the observation group was higher than that of the control group (*P* < 0.05), and the detail information was shown in Table 1.

### 3.2. Comparison of Bone Metabolism Markers between Groups with/without Prebiotics/Probiotics Preparations

The difference in the levels of BGP, total PINP, and *β*-CTX in the two groups before the treatment was not different statistically (*P* > 0.05). After treatment, the levels of BGP, total PINP, and *β*-CTX in both groups were lower than those before treatment, and the levels of BGP, total PINP, and *β*-CTX in the observation group were lower than those in the control group (*P* < 0.05), as shown in Figure 1.

The article "Curative Effect of Prebiotics/Probiotics Preparations Combined with Zoledronic Acid + Calcitriol Regimen on Patients with Primary Osteoporosis and Their Influences on Bone Metabolism Markers" was retracted in 2024. Reasons: signs of a paper mill; suspected computer-generated content; unreliable results or conclusions; lack of ethics approval or compliance.

### 3.3. Comparison of Calcium and Phosphorus Metabolism between Groups with/without Prebiotics/Probiotics Preparations

The level of serum Ca before and after treatment between the two groups was not different statistically (*P* > 0.05). The levels of serum P in both groups after treatment were lower than those before treatment, and the level of serum P in the observation group was lower than that in the control group (*P* < 0.05), as shown in Figure 2.

### 3.4. Comparison of Intestinal Flora between Groups with/without Prebiotics/Probiotics Preparations

The difference in the number of intestinal flora between the two groups before treatment was not statistically significant (*P* > 0.05). The number of *Escherichia coli* after treatment in the two groups were less than that before treatment, and the number of *Escherichia coli* in the observation group was less than that in the control group (*P* < 0.05). The number of bifidobacteria and lactobacilli in the two groups after treatment was more than that before treatment, and the number of bifidobacteria and lactobacilli in the observation group was more than that in the control group (*P* < 0.05), as shown in Figure 3.

### 3.5. The Comparison of Cytokines in Groups with/without Prebiotics/Probiotics Preparations

The difference in the levels of IL-6, TNF-*α*, and IGF-1 between two groups before treatment was not statistically significant (*P* > 0.05). The levels of IL-6 and TNF-*α* in the two groups were lower than those before treatment, and the levels of IL-6 and TNF-*α* in the observation group was lower than those in the control group (*P* < 0.05). The levels of IGF-1 in the two groups after treatment were higher than those before treatment, and the levels of IGF-1 in the observation group was higher than that in the control group (*P* < 0.05), as shown in Figure 4.

## 4. Discussions

POP is a metabolic bone disease, caused by various reasons, which induces a bone density and bone quality decrease as well as increase the risk of fracture. The full name of zoledronic acid is 1-hydroxy-2-(1-imidazolyl) ethylene-1,1-diphosphoric acid monohydrate. The molecular weight of zoledronic acid is 290.11, which is a nitrogen-containing bisphosphonate compound and is a commonly used drug for the treatment of patients with POP. It can act on human bones, inhibit bone resorption by inhibiting osteoclasts, induce their apoptosis, and can regulate osteoblasts and osteoclasts. A cellular transcriptional mechanism reduces osteoclast activity and contributes to the optimization of bone turnover status [6, 7]. Relevant studies have pointed out that zoledronic acid can interfere with the mevalonate metabolic pathway in osteoclasts, induce osteoclast and monocyte precursor cell apoptosis, reduce osteoclast activity, inhibit bone resorption, and play an antibone role of mass loosening [8]. Calcitriol is a 1,25-dihydroxy metabolite of vitamin D3, which is metabolized by liver and kidney hydroxylase. Calcitriol accelerates the formation of new osteoblasts by promoting intestinal calcium absorption and stimulating the activity of osteoblasts in bones. At the same time, calcitriol regulates the transcription mechanism of osteoblasts and osteoclast and reduces the activity of osteoclasts [9, 10]. Some studies have pointed out that abnormal intestinal flora can affect mineral absorption and release serum cytokines to affect bone metabolism [11]. Therefore, we treated the patients with probiotic preparations in this study. Studies have found that combined treatment of probiotics in patients with POP can improve bone metabolism and improve the therapeutic effect. This is mainly related to the fact that probiotics can reduce the release of proinflammatory and osteoclast-related cytokines by improving intestinal flora disturbance [12]. Besides, our results showed the number of *Escherichia coli* in the observation group was less than that in the control group, and the number of bifidobacteria and lactobacilli in the observation group was more than that in the control group, which indicated the gut flora of POP patients was optimized via the prebiotics/probiotics preparations combined with zoledronic acid + calcitriol regimen. The study about the gut microbiota and osteoporosis has raged unabated recently. Gut microbiota contributes to the metabolisms of bones directly or together with nerve, endocrine, and immune systems, which we suppose, is the main factor contributes the improvement of Disorders of bone metabolism in POP patients. For instance, the unbalanced osteogenic and osteoclast responses resulting in osteopenia may be contributed by the unbalanced gut microbiota [7].

The article "Curative Effect of Prebiotics/Probiotics Preparations Combined with Zoledronic Acid + Calcitriol Regimen on Patients with Primary Osteoporosis and Their Influences on Bone Metabolism Markers" was retracted in 2024. Reasons: signs of a paper mill; suspected computer-generated content; unreliable results or conclusions; lack of ethics approval or compliance.

Gut microbes can influence the release of inflammatory factors, resulting in decreased osteoclastogenesis [8, 13]. IGF-1 is an important factor affecting bone metabolism. It can act on bones through endocrine and autocrine pathways, stimulate the differentiation of osteoblasts, and bind to its receptors to participate in the growth and proliferation of osteocytes, which can promote bone formation. IL-6 can regulate the proliferation, differentiation, and apoptosis of osteoblasts through multiple pathways, and can promote the formation of osteoclasts and bone resorption, leading to the occurrence of POP. TNF-*α* can not only act as an inducer to regulate IL-6 secretion but also act on osteoblasts to indirectly activate mature osteoclasts and inhibit osteoclast apoptosis [14]. The levels of IL-6 and TNF-*α* in the observation group was lower than those in the control group, and the levels of IGF-1 in observation group was higher than that in the control group, which indicated that probiotics could be contribute bone metabolism by inhibiting the secretion of proinflammatory factors. Lots of studies have indicates the preparations of probiotic regulates bone metabolism by reducing proinflammatory and osteoclast-related cytokines. For instance, probiotic contributes the formation of vitamin K, which is lip-soluble and enhance the density of bones. The improvement of osteoporosis and decrease in the bone calcium loss is done by in taking probiotic [15]. Calcium and phosphorus are indispensable macroelements in human body, and the metabolism of calcium and phosphorus in hematoma is closely related to bone metabolism. Some scholars have found that serum calcium and phosphorus levels in patients with osteoporosis are significantly abnormal [16]. Some data show that probiotics promote the transfer of calcium in the blood to the bones to form calcium salts, which provide necessary environment for the new bones growth [17]. The results of this study showed that the level of serum P in the observation group was lower than that in the control group, indicating that the calcium and phosphorus metabolism in patients with POP was improved by probiotic preparations, which was fore mostly due to the transfer of calcium and phosphorus into osteoblasts in peripheral blood induced by the probiotics. Additionally, probiotics function in a fine manner to adjust the balance of calcium in the blood.

In conclusion, prebiotic/probiotic preparations combined with zoledronic acid + calcitriol regimen have high efficacy in the treatment of POP, can improve bone metabolism and intestinal flora, and inhibit the release of cytokines in the body.

## Figures and Tables

**Figure 1:** The changes of bone metabolism markers between the two groups with/without prebiotics/probiotics preparations (compared with the same group before the treatment, ^#^*P* < 0.05; compared with the control group, ^*∗*^*P* < 0.05).

**Figure 2:** Comparison of calcium and phosphorus metabolism indexes between groups with/without prebiotics/probiotics preparations (^#^*P* < 0.05 represents comparing with the same group before treatment; ^*∗*^*P* < 0.05 represents comparing with the control group).

**Figure 3:** The differences of intestinal flora between groups with/without prebiotics/probiotics preparations (^#^*P* < 0.05 represents comparing with the same group before treatment; ^*∗*^*P* < 0.05 represents comparing with the control group).

The article "Curative Effect of Prebiotics/Probiotics Preparations Combined with Zoledronic Acid + Calcitriol Regimen on Patients with Primary Osteoporosis and Their Influences on Bone Metabolism Markers" was retracted in 2024. Reasons: signs of a paper mill; suspected computer-generated content; unreliable results or conclusions; lack of ethics approval or compliance.

**Figure 4:** The comparison of cytokines in groups with/without prebiotics/probiotics preparations (^#^*P* < 0.05 represents comparing with the same group before treatment; ^*∗*^*P* < 0.05 represents comparing with the control group).

**Table 1:** Comparison of therapeutic efficacy between groups with/without prebiotics/probiotics preparations (*n*, (%)).

Group	*n*	Significant valid	Effective	Invalid	Total efficiency
Observation group	63	25	34	4	93.65
Control group	63	20	31	12	80.95
*χ*2					4.582
*P* value					0.032

## Data Availability

The raw data supporting the conclusion of this article will be available by the authors without undue reservation.
